# *Haemophilus influenzae* responds to glucocorticoids used in asthma therapy by modulation of biofilm formation and antibiotic resistance

**DOI:** 10.15252/emmm.201505088

**Published:** 2015-05-20

**Authors:** Chris S Earl, Teh Wooi Keong, Shi-qi An, Sarah Murdoch, Yvonne McCarthy, Junkal Garmendia, Joseph Ward, J Maxwell Dow, Liang Yang, George A O’Toole, Robert P Ryan

**Affiliations:** 1 Division of Molecular Microbiology, College of Life Sciences, University of DundeeDundee, UK; 2 Singapore Centre on Environmental Life Sciences Engineering, Nanyang Technological UniversitySingapore, Singapore; 3 School of Microbiology, Biosciences Institute, University College CorkCork, Ireland; 4 Instituto de Agrobiotecnología, CSIC-Universidad Pública Navarra-Gobierno NavarraMutilva, Spain; 5 Centro de Investigación Biomédica en Red de Enfermedades Respiratorias (CIBERES)Madrid, Spain; 6 Division of Molecular Medicine, College of Life Sciences, University of DundeeDundee, UK; 7 Department of Microbiology and Immunology, Geisel School of Medicine at DartmouthHanover, NH, USA

**Keywords:** antibiotic resistance, asthma, biofilm, *Haemophilus influenzae*, steroids

## Abstract

Glucocorticosteroids are used as a main treatment to reduce airway inflammation in people with asthma who suffer from neutrophilic airway inflammation, a condition frequently associated with *Haemophilus influenzae* colonization. Here we show that glucocorticosteroids have a direct influence on the behavior of *H. influenzae* that may account for associated difficulties with therapy. Using a mouse model of infection, we show that corticosteroid treatment promotes *H. influenzae* persistence. Transcriptomic analysis of bacteria either isolated from infected mouse airway or grown in laboratory medium identified a number of genes encoding regulatory factors whose expression responded to the presence of glucocorticosteroids. Importantly, a number of these corticosteroid-responsive genes also showed elevated expression in *H. influenzae* within sputum from asthma patients undergoing steroid treatment. Addition of corticosteroid to *H. influenzae* led to alteration in biofilm formation and enhanced resistance to azithromycin, and promoted azithromycin resistance in an animal model of respiratory infection. Taken together, these data strongly suggest that *H. influenzae* can respond directly to corticosteroid treatment in the airway potentially influencing biofilm formation, persistence and the efficacy of antibiotic treatment.

See also: **J Reidl & E Monsó** (August 2015)

## Introduction

Asthma is a chronic inflammatory condition of the airways, frequently distinguished by abnormal immune responses to environmental antigens and microbes, which leads to recurrent episodes of cough, wheezing and breathlessness (Wenzel, 2006, 2012). An estimated 300 million people worldwide suffer from asthma. Up to 30% of these patients suffer from neutrophilic asthma, which is characterized by substantial increases in airway neutrophils. Chronic colonization by bacteria is evident in the airways of patients with neutrophilic asthma, with *Haemophilus influenzae* being the species most frequently isolated.

Inhaled glucocorticosteroids, through their potent anti-inflammatory action, are the foundation of asthma therapy (Ito *et al*, 2006). However, in a very high proportion of cases, neutrophilic asthmatics respond poorly to glucocorticosteroid treatment (Essilfie *et al*, 2011, 2012). Chronic bacterial infection has been associated with steroid-resistant neutrophilic asthma, although the mechanisms producing treatment resistance in such infections are poorly understood (Beigelman *et al*, 2014). The occurrence of *Haemophilus* spp.*, Streptococcus* spp. or *Moraxella catarrhalis* in the neutrophilic asthmatic airway has been positively correlated with sputum neutrophilia and lower FEV_1_. The presence of *H. influenzae* in particular has been associated with the activation of airway inflammation pathways in those asthmatics with relative steroid resistance (Green *et al*, 2014). *H. influenzae* infection has been shown to contribute in part to allergic airways disease through alterations in IL-17 (Simpson *et al*, 2006; Berry *et al*, 2007). Furthermore, a strong relationship between chronic *H. influenzae* infection and the development of steroid-resistant neutrophilic asthma has been suggested using murine models of ovalbumin (OVA)-induced allergic airway disease (Essilfie *et al*, 2011, 2012). In this model, the combination of infection and allergic airways disease promotes bacterial persistence leading to the development of a phenotype similar to steroid-resistant neutrophilic asthma. These findings indicate that targeting bacterial infection in steroid-resistant asthma may have a therapeutic benefit.

One aspect of the pathogenesis and therapy of neutrophilic asthma that has not received consideration is the potential direct influence of glucocorticosteroids on the behavior of *H. influenzae*. There are no reports of a direct antibacterial action of glucocorticosteroids; nevertheless, an impact on bacterial functions that promote persistence and tolerance to antibiotics might impinge on the efficacy of therapy. In this context, it is noteworthy that the severity of asthma appears to be increased in patients with bacterial infections who have received prolonged therapy with glucocorticosteroids.

Here we have examined the impact of glucocorticosteroid treatment on *H. influenzae* during respiratory infection and neutrophilic asthma, as well as investigating impacts of this therapeutic *in vitro* on *H. influenzae* biology. Using a mouse model of acute infection, we show that the presence of glucocorticosteroids promotes *H. influenzae* persistence without influencing the host inflammatory response. Comparative transcriptional analysis of *H. influenzae* grown under standard laboratory conditions in the absence and presence of beclomethasone revealed that this glucocorticosteroid induces altered expression of genes implicated in biofilm formation and host colonization. Furthermore, the majority of these genes showed similar alterations in expression when transcriptomes of bacteria grown in medium without glucocorticosteroid were compared with those of bacteria isolated from the airway of infected mice. Importantly, many of the *H. influenzae* genes with expression that was responsive to corticosteroid *in vitro* also had altered expression in bacteria within sputum samples from asthma patients undertaking inhaled steroid treatment. In parallel, we examined the influence of glucocorticosteroids on *H. influenzae* behavior by addressing the effects on biofilm formation and resistance to azithromycin, a frontline drug prescribed to asthma patients. Addition of glucocorticosteroids changed the architecture and increased the tolerance to azithromycin of *H. influenzae* biofilms developed in flow cells. Finally, we developed a mutant screen that allowed the identification of a potential role for the RpoE-MclA sigma factor–anti-sigma factor system (HI0628–HI0629) as a mediator of this glucocorticosteroid response. Taken together, these findings indicate that *H. influenzae* can respond directly to glucocorticosteroid treatment in the lung where it may influence biofilm formation, persistence and the efficacy of antibiotic therapy.

## Results

### Glucocorticosteroids promote *H. influenzae* persistence in a mouse model

Mouse models of *H. influenzae* have been rarely reported since it is difficult for this bacterium to infect mice (Vallee *et al*, 1992; Wu *et al*, 1997). Here, we pursued a new mouse model of lung infection in order to determine whether glucocorticosteroids have the ability to modulate *H. influenzae* infection. We used 4-week-old C57BL/6 mice to assess the effects of supplementation of *H. influenzae* with beclomethasone, a model glucocorticosteroid used widely in the clinic (van den Berge *et al*, 2011), on the bacterial load in the lung. Generally, young immature mice are more susceptible to bacterial infection than fully grown mice. In addition, the mice were pretreated intraperitoneally with cyclophosphamide to induce granulocytopenia. When cyclophosphamide-pretreated mice were intranasally inoculated with 1 × 10^9^ CFU of *H. influenzae*, the bacteria resided in the lungs of the mice at more than 10^5^ CFU for up to 3–4 days post-inoculation.

Next, the cyclophosphamide-treated C57BL/6 mice were infected with *H. influenzae* and treated by inhaling PBS with or without 50 μM beclomethasone, a clinically relevant dose based on the weight of the mice used (Daley-Yates *et al*, 2001). The lung and spleen bacterial load was determined at 1, 3, 5 or 7 days post-infection. C57BL/6 mice infected with *H. influenzae* with PBS cleared almost all bacteria from the lungs within 5 days (Fig1A). However, with the addition of beclomethasone, bacteria were still present in substantial numbers at 7 days (Fig1A), with ∼1,000-fold more bacteria present in the beclomethasone-treated mice versus control. Similar patterns were seen in the bacterial loads in the spleen, where after 7 days the numbers of bacteria in beclomethasone-treated mice were significantly higher (∼1.5 log higher) than in untreated mice (Fig1B). To extend this study, we also examined the influence of mometasone and prednisolone, two other glucocorticosteroids in clinical use, on *H. influenzae* survival in the cyclophosphamide-mouse model. Treatment with prednisolone (50 μM) gave a similar increased persistence phenotype as was observed for beclomethasone treatment (Supplementary Fig S1). Mometasone (50 μM) also appeared to promote *H. influenzae* persistence, although its influence was considerably less than the other two steroids tested.

**Figure 1:** Administration of corticosteroids promotes the persistence of *H. influenzae* in mice A–D C57BL/6 mice were infected with *H. influenzae* in PBS with or without supplementation with beclomethasone. Animals were killed at 1, 3, 5 and 7 days after infection, and 10-fold serial dilutions of the lung homogenates (A) and spleen homogenates (B) were plated to determine the bacterial load. Airway inflammation represented by total and differential cell counts in bronchoalveolar lavage fluid (BALF). The number of total leukocytes and in particular of neutrophils, monocytes and lymphocytes recruited in the airways was analyzed in BALF after day 3 (C) and day 7 (D) of infection. Data information: Values represent the mean ± standard deviation (SD). The data are pooled from three independent experiments. Statistical significance by two-tailed Student’s *t*-test is indicated: *P < 0.05, **P < 0.01.

The effects of beclomethasone on *H. influenzae* persistence were also examined in C57BL/6 mice that did not receive the cyclophosphamide treatment. The same trend was observed where beclomethasone treatment enhanced *H. influenzae* persistence in the airway, although in this case, no dissemination to the spleen was seen (Supplementary Fig S2). Taken together, these data indicate that treatment with beclomethasone enhanced *H. influenzae* persistence in the airway and systemically in this model of infection.

Numerous previous studies have demonstrated *H. influenzae* infection of the murine airway induces the recruitment of leukocytes and other inflammation markers, which mirrors in part what is seen in a clinical setting (Hansen *et al*, 1988; Essilfie *et al*, 2011, 2012). In the current study, the inflammatory response of challenged mice was examined in terms of total leukocyte recruitment in the airways (see Materials and Methods). In the first set of experiments, mice were pre-treated with cyclophosphamide. At 3 days post-infection, the cell numbers that influx into the airways (including neutrophils, lymphocyte and eosinophils) were similar in beclomethasone-treated mice and mice that were treated with PBS only (Fig1C). By 7 days post-infection, however, neutrophil numbers in the mice treated with beclomethasone remained at the level seen at 3 days and were significantly higher than those seen in PBS alone (Fig1D). In contrast, overall lymphocyte numbers were similar in mice treated with beclomethasone compared with mice treated with PBS alone (Fig1D). The effects of beclomethasone on the inflammatory response induced by *H. influenzae* in C57BL/6 mice that did not receive the cyclophosphamide treatment were also examined. In this case, more neutrophils were recruited on day 3 as with the cyclophosphamide-treated mice (Supplementary Fig S2), but this elevation returned to normal levels by day 4.

The observed continued recruitment of neutrophils at day 7 in the cyclophosphamide-mouse model of *H. influenzae* infection was unexpected. However, this observation is not unprecedented in the clinical setting; examination of neutrophilic asthma patients showed neutrophil numbers increase in those patients undergoing inhaled corticosteroid treatment (see Simpson *et al*, 2006). Overall, our results suggest that the presence of beclomethasone increases the capacity of *H. influenzae* to persist in mice but these findings do not establish whether this is a direct effect of the glucocorticosteroid on the bacteria or whether this is an indirect effect, mediated through an influence on the host, including recruitment of immune cells.

### Glucocorticosteroids induce specific changes in *H. influenzae* gene expression in culture

As an approach to understanding the possible direct influence of glucocorticosteroids on *H. influenzae*, we examined the impact of beclomethasone on gene expression of bacteria using high-throughput cDNA sequencing techniques. For these experiments, bacteria were grown in complex sBHI medium, which is brain–heart infusion medium supplemented with hemin and NAD (see Materials and Methods). RNA was derived from bacteria grown in the presence and absence of beclomethasone (50 μM) and, following rRNA depletion, the remaining RNA was fragmented, reverse-transcribed into cDNA and sequenced using the Illumina platform. Between 20 and 30 million reads were derived from each sample, which were aligned to non-rRNA sequences in the *H. influenzae* genome, comprising the 1,788 annotated ORFs (Supplementary Table S1). The correlation of technical replicates was very high, suggesting that variations introduced during library construction and sequencing do not significantly contribute to differences in gene expression between samples. A total of 61 genes were significantly differentially expressed by at least threefold (P_adj_ < 1 × 10^−5^) during growth of *H. influenzae* in sBHI in the presence or absence of beclomethasone (see Materials and Methods). Of the 61 genes regulated by beclomethasone, 29 genes were up-regulated and 32 genes were down-regulated (Fig2A and B and Supplementary Table S2).

**Figure 2:** *H. influenzae* genes differentially regulated during growth in complex media and during lung infection in the presence of corticosteroids A Venn diagram showing the overlap of *H. influenzae* genes whose expression is up-regulated or down-regulated by the presence of corticosteroids in sBHI medium (*in vitro*) or in the mouse model of infection (*in vivo*). Genes that are divergently regulated in these conditions are not depicted in this Venn diagram but can be found in the complete RNA-Seq dataset detailed in Supplementary Table S2.

B COG map detailing significantly enriched or scarce functional categories expressed *in vitro* and *in vivo* during the presence of corticosteroids.

C, D Comparison of relative fold changes between RNA-seq and qRT–PCR results *in vitro* (C) and *in vivo* (D) in the presence of corticosteroids. All qRT–PCR results were normalized using the *Ct*s obtained for the 16S rRNA amplifications run in the same plate. The relative levels of gene transcripts are determined from standard curves. Values given are the mean and standard deviation of triplicate measurements (three biological and three technical replicates).

Those genes whose expression was increased by beclomethasone treatment included those with protein products involved in adaptive responses such as iron uptake (HI0994), biofilm formation (HI1344), stress response (HI0628) and antimicrobial resistance (HI1275) as well as the *yfe* operon (*HI0359–HI0362*), which encodes an ABC transporter putatively involved in metal ion uptake and previously implicated in *H. influenzae* virulence regulation, adherence to host cells and host immune evasion (Whitby *et al*, 2006; Jalalvand *et al*, 2013; Su *et al*, 2013).

The effect of beclomethasone on the level of transcript was validated by quantitative reverse-transcription polymerase chain reaction (qRT–PCR). The genes selected for these analyses represented those from diverse functional classes with some previously implicated in virulence and biofilm regulation in *H. influenzae* with a fold change of three or higher (Fig2C). Importantly, this subset of those genes that showed a response to beclomethasone showed a similar alteration in expression when *H. influenzae* was cultured in the presence of prednisolone, another glucocorticosteroid taken by asthmatics (Supplementary Figs S3 and S4). In contrast, many of these genes showed no alteration in expression in response to dehydroepiandrosterone, an unrelated steroid that is found abundantly in human tissue (Supplementary Fig S3).

### Genes showing specific changes in expression during *H. influenzae* infection include a subset that is influenced by glucocorticosteroids in culture

The effects of glucocorticosteroids on gene expression of *H. influenzae* in culture raised the issue of whether similar alterations in gene expression occur in the mouse model treated with glucocorticosteroids. As with other opportunistic pathogens, *H. influenzae* modulates its gene expression upon colonization of its mammalian host. To gain understanding of this adaptation of *H. influenzae* to the host environment (in the presence of beclomethasone treatment), we systematically cataloged the transcriptomes of bacteria grown *in vivo*, using high-throughput cDNA sequencing techniques. RNA was derived from organisms isolated directly from the lung homogenates of infected mice and, following rRNA depletion, the remaining RNA was fragmented, reverse-transcribed into cDNA and sequenced. Illumina-based RNA-seq was used for the characterization of bacteria within the lung tissue, which reach densities of 10^5^ CFU/ml. We chose to profile the infection 3 days post-inoculation because this represents the midpoint of the trajectory of the infection.

A total of 35–40 million reads were derived from murine samples and were aligned to non-rRNA sequences in the *H. influenzae* genome (Supplementary Table S1). To identify genes that are differentially expressed during murine infection and in sBHI medium with or without glucocorticosteroid, we compared the RNA-seq data for these conditions using DESeq, a differential expression analysis package for RNA-seq data that presumes that abundance of reads can be modeled by a negative binomial distribution (An *et al*, 2013). These analyses revealed that expression of 129 (7.2%) of the 1,788 annotated *H. influenzae* ORFs was significantly altered (> 3-fold, P_adj_ < 1 × 10^−5^) in the mouse model of infection by comparison with bacteria grown in culture without glucocorticosteroids; expression of 58 genes (3.2%) was up-regulated, whereas expression of 71 genes (4.0%) was down-regulated (Fig2A and B and Supplementary Table S2).

Comparison of these alterations in the transcriptome with those induced by the presence of beclomethasone in culture revealed a significant overlap (Fig2A and Supplementary Table S2). Nevertheless, a large number of genes (*n* = 82) whose expression is altered in bacteria in the host are not regulated by glucocorticosteroids in culture, consistent with the contention that these are responses of *H. influenzae* to other aspects of the host environment. While the majority of these differentially expressed genes were annotated as hypothetical proteins, several have recently been shown to encode factors required by *H. influenzae* for growth and/or colonization of the host. These included *HI0174* (*mnmA*), *HI0274* (*gltX*), *HI0479* (*atpD*), *HI0629* (*mclA*), *HI1547* (*aroG*) and *HI1548* (*lolE*) (Gawronski *et al*, 2009). Additional regulated genes encoded factors that have been previously reported to contribute to *H. influenzae* virulence: *HI1544* which encodes a NAD(P)H oxidoreductase and *HI1707* which encodes the sensor kinase, FirS (Steele *et al*, 2012).

To assess the reliability of RNA-seq data in determining the relative abundances of individual transcripts in the presence of beclomethasone, we used the same total RNA samples determined by qRT–PCR: the mRNA levels of five up-regulated genes (*HI0075*, *HI0095*, *HI0628*, *HI1275* and *HI1677*) and four down-regulated genes (*HI0127*, *HI0811*, *HI1177* and *HI1431*) (Fig2D). The ratios of the transcripts from samples determined by RNA-seq to those obtained by qRT–PCR were in concordance.

### Transcript levels of glucocorticosteroid-responsive *H. influenzae* genes in sputum from asthma patients

The above findings suggest that glucocorticosteroids may influence the expression of specific *H. influenzae* genes in asthma patients. In order to test this hypothesis, the transcript level of three corticosteroid-responsive genes (*HI0359, HI0628* and *HI0994*) was established by qRT–PCR on sputum samples collected from twenty-four asthma patients. A comparison of the demographics and asthma characteristics of these patients are shown in Table1. There were no significant differences in gender, smoking history (defined as % current and past smoker), obesity (defined as BMI ≥ 30 kg/m^2^), nasal disease, atopy and serum IgE. All patients were taking standard inhaled glucocorticosteroid therapy using beclomethasone or mometasone routinely.

**Table 1:** Summary of bacteria identified by culturing and the detection of bacterial gene transcription in the sputum from asthma patients

Sample no.	Age (y) and sex	FEV1%	Inhaled steroid treatment^a^	Detected bacterial strains^b^	mRNA level^c^		
					*HI0359*	*HI0628*	*HI0994*
S1	27 (M)	26	Bec	Hi, Sp	24.9 (0.4)	4.4 (0.9)	7.1 (0.2)
S2	26 (F)	32	Bec	Hi, Pa, Sa, MRSA, Ko, Sm	18.9 (0.4)	4.3 (0.6)	6.9 (0.6)
S3	26 (F)	29	Bec	Hi, Pa, Sa, Ko, Sm	12.8 (0.1)	4.4 (0.2)	6.7 (0.3)
S5	24 (M)	33	Bec	Hi, Sm, Mc	9.3 (0.9)	4.6 (0.8)	6.4 (0.2)
S8	22 (F)	23	Bec	Hi, Pa, Sa, Ko, Sm	8.6 (0.2)	7.8 (0.2)	5.2 (0.2)
S9	26 (M)	24	Bec	Hi, Pa, Sa, Ko, Sm	8.5 (0.1)	4.7 (0.8)	5.1 (0.1)
S10	25 (M)	33	Bec	Hi, Pa, Sm, Mc	8.2 (0.3)	5.1 (0.4)	5.0 (0.7)
S12	26 (F)	31	Bec	Hi, Pa, Sa, Ko, Sm	7.2 (0.3)	4.2 (0.6)	4.7 (0.4)
S13	26 (F)	30	Bec	Hi, Pa, Sa, MRSA, Ko, Sm	6.3 (0.1)	4.0 (0.6)	4.2 (0.2)
S14	26 (F)	27	Bec	Hi, Pa, Sa, Ko, Sm, Sp	6.2 (0.3)	3.0 (0.7)	4.1 (0.5)
S15	25 (F)	26	Bec	Hi, Ko, Sm	6.0 (0.2)	3.3 (0.4)	3.9 (0.8)
S16	23 (M)	29	Bec	Hi, Pa, Sa, Ko, Sm	5.2 (0.3)	2.9 (0.7)	3.5 (0.6)
S18	25 (M)	32	Bec	Hi, Pa, Sa, Ko, Sm	4.7 (0.7)	2.5 (0.6)	3.4 (0.8)
S22	26 (M)	26	Bec	Hi, Pa, Sa, Ko, Sm	4.5 (0.9)	2.3 (0.6)	3.4 (0.7)
S24	27 (M)	28	Bec	Hi, Pa, Sa, Ko, Sm	3.9 (0.4)	2.2 (0.4)	3.3 (0.9)
S6	23 (M)	30	Mom	Hi, Pa, Sa, Ko, Sm	3.7 (0.8)	2.9 (0.1)	2.9 (0.3)
S7	22 (M)	27	Mom	Hi, Ko, Sm, Sp	2.5 (0.2)	2.3 (0.6)	2.6 (0.2)
S17	26 (F)	31	Mom	Hi, Ko, Sm	2.5 (0.1)	2.8 (0.2)	2.5 (0.2)
S19	26 (F)	30	Mom	Hi, Pa, Sa, Ko, Sm	2.5 (0.5)	2.7 (0.5)	2.2 (0.6)
S23	25 (F)	31	Mom	Hi, Ko, Sm	2.4 (0.6)	2.1 (0.5)	2.0 (0.9)
S11	26 (M)	30	Bec	Pa, Sa, Ko, Sm	N/A	N/A	N/A
S20	27 (F)	30	Bec	Pa, Sa, Ko, Sm	N/A	3.1 (0.5)	N/A
S21	26 (F)	29	Mom	Pa, Sa, Ko, Sm	2.0 (0.4)	N/A	N/A
S4	26 (M)	30	N/A	Pa, Sa, MRSA, Ko, Sm	N/A	N/A	N/A

a Current steroid treatment, Bec (beclomethasone) or Mom (mometasone).

b Abbreviations of microbes identified by culture-based methods: Hi (*H. influenzae*), Pa (*Pseudomonas aeruginosa*), Sa (*Staphylococcus aureus*), Ko (*Klebsiella oxytoca*), Sm (*Stenotrophomonas maltophilia*)*,* MRSA (methicillin-resistant *S. aureus*), Sp (*Streptococcus pneumoniae*) and Mc (*Moraxella catarrhalis*).

c Fold change relative to 16S RNA gene expression (standard deviation).

Inhaled beclomethasone is prescribed much more frequently (in 90% of cases) than mometasone, probably because it is effective but of lower cost than mometasone (Friedman *et al*, 2010). However, mometasone only needs to be administered once every 24 h, whereas beclomethasone is administered two or three times in the same period. The clinical choice between beclomethasone and mometasone is informed by cost, administration frequency as well as past experience (Friedman *et al*, 2010).

Patients had a significant load of pathogenic bacteria in their sputum as detected by culture methods. The bacteria detected included *H. influenzae, Pseudomonas aeruginosa, Staphylococcus aureus,* methicillin-resistant *S. aureus* (MRSA*), Streptococcus pneumoniae, Moraxella catarrhalis, Achromobacter xylosoxidans, Klebsiella oxytoca* and *Stenotrophomonas maltophilia* (Table1). *H. influenzae* was identified in 20 of the 24 sputum samples with *P. aeruginosa* and *S. aureus* being even more commonly found. All patients had more than one bacterial species cultured.

Total RNA was isolated from the 24 sputum samples obtained from these asthma patients. Contaminating DNA was degraded, total RNA was quantified, and equal amounts were subjected to qRT–PCR. Overall, 20 of the 24 sputum samples from patients tested positive for the expression of the selected corticosteroid-responsive genes *HI0359, HI0628* and *HI0994*. There was a direct correlation between the presence of a qRT–PCR amplicon and the presence of *H. influenzae* in sputum as revealed by culture but no correlation with the presence of any other pathogenic bacteria. Notably, the transcript level of these target genes was increased in patients who were currently using beclomethasone compared to those who were using mometasone (Table1).

### Clinical isolates of *H. influenzae* retain the ability to respond to glucocorticosteroid

Although an elevated level of expression of corticoid-responsive genes in *H. influenzae* strains in sputum from asthma patients is consistent with a direct response to beclomethasone, the findings do not exclude the possibility that clinical isolates have intrinsically higher levels of expression of these genes. To address this issue, the ability of a panel of seven *H. influenzae* clinical isolates to respond to glucocorticosteroids was assessed by measurement of the expression of *yfe* operon (*HI0359–HI0362*) and *HI0628* and *HI0994* by qRT–PCR. Addition of beclomethasone or prednisone to the *H. influenzae* isolates led to the up-regulation of *yfe* operon (*HI0359–HI0362*) and *HI0628* and *HI0994* in all strains, although to varying degrees (Supplementary Table S3). However, the level of alteration in expression in response to mometasone was considerably reduced (Supplementary Table S3). Taken together, the findings indicate that clinical isolates of *H. influenzae* retain the ability to respond to beclomethasone.

### Identities of genes that mediate the response of *H. influenzae* to glucocorticosteroids

We next sought to understand the mechanism by which beclomethasone impacts bacterial gene expression. As outlined above, the addition of beclomethasone to *H. influenzae* cultures led to increased expression of *HI1677*, which encodes an iron–sulfur cluster repair protein (Fig2D). This observation formed the basis of a screen for genes involved in the beclomethasone response. A reporter strain was constructed in which the *luxCDABE* genes were put under control of the *HI1677* promoter in the wild-type background (see Materials and Methods). This *HI1677*::*lux* reporter strain was subjected to insertional mutagenesis using a kanamycin resistance (Kan^R^) cassette as described in the Materials and Methods. A panel of approximately 4,000 mutants was screened for altered bioluminescence in the presence of beclomethasone (50 μM). Initially, 34 mutants that demonstrated altered expression of the reporter fusion were isolated, and following a rescreening to reduce false negatives, 19 candidates with altered response were identified.

The sites of Kan^R^ cassette insertion for the non-responsive mutants were mapped to the genome of *H. influenzae* by polymerase chain reaction (PCR) and sequencing of amplicons (see Materials and Methods). Southern blot analysis confirmed that only a single copy of the cassette was inserted into the chromosome in these non-responsive mutants. Insertion sites, which were all different, were mapped to seven genetic loci with three genes found more than once. None of the mutants showed impaired growth in complex or minimal media, suggesting that the altered response to corticosteroid could not be attributed to differences in growth (Table2).

**Table 2:** Location of transposon insertions that influence activation of the *H. influenzae HI1677*::*lux* reporter by beclomethasone

Disrupted gene^a^	Polar effect possible^b^	Hits of individual transposon mutants^c^	Gene product
HI0334	Y	2	GTP pyrophosphokinase, RelA
HI0628	Y	1	RNA polymerase sigma factor, RpoE
HI0910	N	1	Mutator protein, MutT
HI0999	Y	2	Ribonuclease P, RnpA
HI1275	Y	1	Tellurite resistance protein, TehB
HI1501	N	1	Hypothetical protein
HI1605	Y	1	Hypothetical protein

a None of these gene disruptions affect bacterial growth in complex media and minimal media.

b Possibility of Tn5 insertion affecting expression of other (downstream) genes. Y: yes; N: no.

c Number of different Tn5 insertion mutations mapped to the same gene.

Mutations were found in several genes encoding proteins involved in stress response (such as *HI0999* and *HI1275*), in genes encoding hypothetical protein (*HI1501*) and in genes encoding regulatory proteins including RpoE (*HI0628*). Other insertions were found in genes that have been implicated in adaptation of *H. influenzae* to infection of the murine lung (*HI0334*, *HI0910* and *HI1605*). RpoE (also known as σ^E^) belongs to the extracytoplasmic function (ECF) family of sigma factors (Craig *et al*, 2001, 2002). These ECF sigma factors, often functioning together with a membrane-associated anti-sigma factor, act to transduce signals perceived outside the cell membrane into a transcriptional response. On the basis of their putative action in the perception of extracellular signals, subsequent work focused on the potential role of the RpoE (HI0628) in the response of *H. influenzae* to glucocorticosteroids.

### RpoE regulates the expression of a subset of the genes influenced by glucocorticosteroids

Previous studies demonstrated that *rpoE* (*HI0628*) is part of an extracytoplasmic stress operon that is required for intracellular survival of *H. influenzae* (Craig *et al*, 2001, 2002). *HI0629* (*mclA*), which is immediately downstream of *HI0628*, encodes an anti-sigma factor that modulates the action of RpoE. To examine the extent of the overlap between those genes regulated by glucocorticosteroids and those regulated by *rpoE* or *mclA*, we first established the effect of deletion of *rpoE* or *mclA* on the global gene expression patterns. The transcriptomes of *rpoE* and *mclA* deletion mutants (constructed as described in Materials and Methods) were compared with the wild-type *H. influenzae* using RNA-seq.

Comparative transcriptome profiling of the *rpoE* deletion mutant and the wild-type parent established that expression of 68 genes was significantly influenced (> 3-fold change) by the loss of the sigma factor (Fig3A, Supplementary Table S2). This analysis revealed that HI0628 controls expression of genes associated with a range of biological functions that include bacterial motility and attachment, stress tolerance, virulence, regulation, transport, multidrug resistance, detoxification and signal transduction. Genes associated with virulence and the formation of biofilms that are regulated by HI0628 include *yfe* operon (*HI0359–HI0362*), *argR* (*HI1209*) and *potD* (*HI1344*).

**Figure 3:** Comparative transcriptome profiling of the effects of the addition of corticosteroid or mutation of *rpoE* or *mclA* on gene expression in *H. influenzae* A Venn diagrams showing the overlap of *H. influenzae* genes whose expression is influenced by the mutation of *rpoE* or *mclA* or by the presence of corticosteroids in sBHI medium (*in vitro*) or in the mouse model of infection (*in vivo*). The complete set of regulated genes is depicted in Supplementary Table S2.

B, C Comparison of relative fold changes between RNA-seq and qRT–PCR results for *rpoE* and *mclA* mutants (B) and the *rpoE* and the addition of corticosteroid to wild-type *H. influenzae* (C). All qRT–PCR results were normalized using the *Ct*s obtained for the 16S rRNA amplifications run in the same plate. The relative levels of gene transcripts are determined from standard curves. Values given are the mean and standard deviation of triplicate measurements (three biological and three technical replicates).

Inactivation of *mclA* led to significant alteration in the expression of 40 genes, the majority encoding hypothetical proteins. MclA and RpoE influenced expression of many of the same genes. For the majority of these genes, regulation was in opposite direction, which is consistent with the notion that MclA is a negative regulator of RpoE activity (Fig3B). Nevertheless, RpoE and MclA regulated a small number of genes in the same direction (Fig3B). The alteration in expression as revealed by the RNA-seq analysis was confirmed for selected genes by qRT–PCR (Fig3B).

Comparisons of the effect on the transcriptome profile of *rpoE* (*HI0628*) mutation and the addition of exogenous corticosteroid revealed a number of genes (*n* = 66) whose expression appeared to be co-regulated (Fig3A, Supplementary Table S2). Several transcriptional changes in co-regulated genes caused by *rpoE* mutation and corticosteroid addition to *H. influenzae* were confirmed by qRT–PCR (Fig3C). As outlined above, MclA influenced many of these genes in the opposite directions to RpoE. Taken together, these findings are consistent with the contention that the RpoE–MclA system is modulated by glucocorticosteroids leading to altered expression of a specific subset of genes; however, our data also indicate that a subset of genes modulated by glucocorticosteroid addition are impacted independently of RpoE.

### Glucocorticosteroids can influence biofilm formation and antibiotic tolerance by *H. influenzae in vitro*

The influence of glucocorticosteroids on expression of genes implicated in biofilm formation and antibiotic tolerance in *H. influenzae* prompted us to examine the effect of beclomethasone on these phenotypes. For these experiments, *H. influenzae* was grown in μ-well chambers with sBHI medium and the bacteria were visualized with SYTO9 (see Materials and Methods). When grown alone, *H. influenzae* formed flat biofilms with little heterogeneity (Fig4A(i)). The addition of 1 μM glucocorticosteroid to the sBHI medium promoted the development of a biofilm with a similar biomass to the bacteria grown without addition, although the structure showed less dense packing of cells (Fig4A(ii)). This alteration in biofilm formation was not seen when dehydroepiandrosterone, a non-corticosteroid, was used in the assay (Supplementary Fig S5).

**Figure 4:** Addition of corticosteroids affects biofilm formation and antibiotic tolerance of H. influenzae *H. influenzae* biofilms were developed after 24 h in μ-well chambers in sBHI medium with and without corticosteroid and were then treated with the antibiotic azithromycin as specified. (i) *H. influenzae* wild-type with DMSO (solvent control); (ii) *H. influenzae* wild-type treated with 1 μM beclomethasone (BEC); (iii) *H. influenzae* wild-type treated with 150 μg/ml azithromycin (AZO); and (iv) *H. influenzae* wild-type treated with 1 μM beclomethasone (BEC) and 150 μg/ml azithromycin (AZO). For these experiments, *H. influenzae* was visualized with SYTO9 (green strain), as described in Materials and Methods. Scale bars = 20 μm. Images shown are representative of 12 images from five independent experiments.

The biofilm biomass after treatments was quantified using COMSTAT. Data are presented as the average of five replicates, with error bar representing the standard deviation of the data. Statistical significance by two-tailed Student’s *t*-test is indicated: **P < 0.01.

Previous studies have shown that *H. influenzae* biofilms cultured in sBHI medium are extremely tolerant to antibiotic treatment, mimicking to an extent what is seen during infection (Swords *et al*, 2004; Starner *et al*, 2008). To examine the influence of beclomethasone on antibiotic tolerance, *H. influenzae* biofilms generated in the presence and absence of 1 μM beclomethasone for 24 h were treated with azithromycin, an antibiotic often prescribed to asthma patients, at 150 μg/ml, which is a concentration measured in the lungs of patients (Starner *et al*, 2008). After 24 h of growth, the presence of azithromycin had substantially inhibited biofilm formation, with significantly decreased biofilm biomass and maximal thickness compared to the untreated control (Fig4A(iii) and B). The presence of 1 μM beclomethasone decreased the effect of azithromycin on *H. influenzae* biofilms, as indicated by a lesser effect on biofilm biomass (Fig4A(iv) and B). In contrast, the addition of dehydroepiandrosterone, which is not a glucocorticoid, did not alter the effect of azithromycin on *H. influenzae* biofilms (Supplementary Fig S5). These data suggest that glucocorticoid treatment of *H. influenzae* biofilms results in an increase in the tolerance to azithromycin. Importantly, *H. influenzae* strains grown planktonically in the presence and absence of beclomethasone showed no difference in tolerance to azithromycin (Supplementary Fig S6).

The role of RpoE and MclA on *H. influenzae* biofilm formation and antibiotic tolerance was also investigated by the examination of biofilm grown in μ-well chambers with sBHI medium. The *rpoE* and *mclA* mutant showed development of a biofilm with a similar biomass to the wild-type, although the bacteria within the structure were slightly less densely packed (Fig5A(i–iii)). Interestingly, mutation of *rpoE* led to the *H. influenzae* biofilm being more tolerant to azithromycin treatment compared to wild-type (Fig5A(iv-v) and B, Supplementary Fig S7). Similarly, mutation of *mclA* mutant led to an increase in azithromycin tolerance (Fig5B, Supplementary Fig S7). Complementation restored these phenotypes toward wild-type (Supplementary Fig S7). To determine whether *rpoE* has a similar influence in clinical isolates of *H. influenzae*, the gene was disrupted in two clinical isolates and mutants were assessed for alterations in phenotype. In these two strains, mutation of *rpoE* led to an enhanced azithromycin tolerance (Supplementary Fig S8), indicating a similar role for RpoE in both clinical and laboratory strains.

**Figure 5:** Mutation of genes encoding RpoE (HI0628) and MclA (HI0629) has similar effects on biofilm formation and antibiotic tolerance in H. influenzae Biofilms of different *H. influenzae* strains were developed after 24 h in μ-well chambers in sBHI medium and were then treated with the antibiotic azithromycin as specified. (i) *H. influenzae* wild-type; (ii) *rpoE* (*HI0628*); (iii) *mclA* (*HI0629*); (iv) *H. influenzae* wild-type treated with 150 μg/ml azithromycin; (v) *rpoE* (*HI0628*) treated with 150 μg/ml azithromycin; (vi) *mclA* (*HI0629*) treated with 150 μg/ml azithromycin. For these experiments, *H. influenzae* was visualized with SYTO9 (green strain), as described in Materials and Methods. Scale bars = 20 μm. Images shown are representative of 12 images from five independent experiments.

The biofilm biomass after treatments was quantified using COMSTAT. Data are presented as the average of five replicates, with error bars representing the standard deviation of the data. Statistical significance by two-tailed Student’s *t*-test is indicated: **P < 0.01.

### Glucocorticosteroids reduce the efficacy of azithromycin treatment against *H. influenzae* colonization in the mouse airway

There have been only a handful of reports addressing the effectiveness of antibiotic treatment against *H. influenzae* during respiratory infection (Vallee *et al*, 1992; Sekiya *et al*, 2008). Therefore, to build on our observations that beclomethasone increases the capacity of *H. influenzae* to tolerate azithromycin in an *in vitro* model, we wished to assess the effect of beclomethasone on the efficacy of azithromycin treatment in a mouse model of infection.

Using a slight modification of the mouse model described above (see Materials and Methods), the C57BL/6 mice were infected with 1 × 10^8^ CFU of *H. influenzae* and treated by inhaling PBS with or without 50 μM beclomethasone. Azithromycin was administered at a concentration of 100 mg/kg/24 h, a dose reported by several studies (Azoulay-Dupuis *et al*, 1991; Girard *et al*, 2005). The lung and spleen bacterial load was determined 3 days post-infection. C57BL/6 mice infected with *H. influenzae* with PBS exhibited considerable colonization (Fig6A and B). Azithromycin appeared to be very effective in eradicating *H. influenzae* from mice treated with PBS alone (Fig6A and B). However, with the addition of beclomethasone, bacteria appear to be present even after the mice had received 3 days of azithromycin treatment (Fig6A and B).

**Figure 6:** Corticosteroid treatment affects *H. influenzae* clearance by antibiotic treatment in the mouse airway A, B Mice infected intranasally with 1 × 10^8 ^CFU *H. influenzae* and treated by inhaling PBS with or without 50 μM beclomethasone. Azithromycin was administered at a concentration of 100 mg/kg/24 h, daily for 3 days after infection. On day 3–4 after infection, the mice were harvested, and bacterial loads were determined in lung (A) and spleen (B) homogenates. Values represent the mean ± standard deviation (SD). The data are pooled from three independent experiments. Statistical significance by two-tailed Student’s *t*-test is indicated: *P < 0.05, **P < 0.01.

The role of RpoE in modulation of the efficacy of azithromycin treatment during airway infection of mice was also investigated by studies of the clearance of the *rpoE* mutant. The *rpoE* mutant showed similar persistence during azithromycin treatment as the wild-type *H. influenzae* with added beclomethasone (Fig6A and B). Addition of beclomethasone to the *rpoE* mutant had no additional effect in C57BL/6 mice. These results suggest that the presence of beclomethasone increases the capacity of *H. influenzae* to persist in wild-type mice undergoing azithromycin treatment and that this persistence effect is modulated by RpoE.

## Discussion

The work in this paper suggests that glucocorticosteroids such as beclomethasone have a direct and specific effect on *H. influenzae*, influencing expression of a subset of genes that underpin alterations in phenotypes, which include biofilm architecture and tolerance to antibiotic treatment *in vitro*. In a mouse model, beclomethasone increased the persistence of *H. influenzae* and reduced the efficacy of azithromycin in clearing the infection. These latter findings are consistent with previous observations using an infant mouse model of bacterial meningitis, where dexamethasone was shown to enhance the persistence of *H. influenzae* in blood and cerebral spinal fluid from mice undergoing treatment with the oral antibiotic cefuroxime (Rodriguez *et al*, 1991). The effects of glucocorticosteroid on the behavior of *H. influenzae* in mice may also be mediated by influences on the host as well as by direct effects on the bacterium. Indeed, it is now appreciated that the action of glucocorticoids can be more complex than simply acting as anti-inflammatory agents (reviewed in Cruz-Topete & Cidlowski, 2015). For example, glucocorticoids synergistically enhance the expression of TLR2 by *H. influenzae* in cultured human epithelial cells (Shuto *et al*, 2002).

Extrapolations from these models of infection to the asthma airway should be made cautiously; nevertheless, several lines of evidence support the notion that beclomethasone affects the behavior of *H. influenzae* in the asthma airway. Analysis of sputum taken from patients with asthma demonstrated elevated transcript level of three glucocorticosteroid-responsive genes (*HI0359, HI0628* and *HI0994*), which was strongly correlated with the use of beclomethasone in patients colonized by *H. influenzae* (Table1). In contrast, the transcript level of these target genes was lower in patients who were currently using mometasone (Table1). Furthermore, testing of a panel of *H. influenzae* clinical isolates showed that each had a similar response to beclomethasone as the model strain in altered transcription of *HI0359, HI0628* and *HI0994* (Supplementary Table S3). These findings indicate that these clinical isolates do not have an intrinsically higher level of expression of these target genes and support the conclusion that the pattern of gene expression of bacteria in sputum is, at least in part, a response to beclomethasone. These similarities to the behavior of the model strain further suggest that the presence of beclomethasone makes a contribution to the enhanced ability of *H. influenzae* to persist during antibiotic treatment for asthma.

Glucocorticosteroid treatments of asthma patients are associated with anti-inflammatory properties, but this contrasts with the response observed in our mouse model following bacterial infection. In challenged mice, glucocorticosteroid treatment showed similar increase in neutrophils and other immune cells comparable to mice that did not receive treatment. The anti-inflammatory activities of glucocorticosteroids in this situation may be counterbalanced *in vivo* by enhanced bacterial persistence. Furthermore, as mentioned above, glucocorticoids can have actions other than as anti-inflammatory agents, for example, in synergistic enhancement of the expression of TLR2 by *H. influenzae* (Shuto *et al*, 2002).

The detailed mechanisms by which beclomethasone exerts its influence on *H. influenzae* gene expression and phenotypes such as biofilm formation and antibiotic tolerance remain obscure. Currently, no glucocorticosteroid receptors have been identified in bacterial cells. Our mutant screen coupled with comparative transcriptomics indicates that some of the effects of beclomethasone may be exerted through an influence on the regulation of the ECF sigma factor RpoE and its anti-sigma factor MclA. In the *H. influenzae* genome, *rpoE* is organized in an operon with *mclA* (also known as *rseA*) and *rseB* (*HI0630*). Homologous genes are present and organized in the same manner in the *E. coli* genome. In *E. coli*, RpoE is normally sequestered to the cytoplasmic face of the inner membrane by an anti-sigma factor, RseA, which interacts with the periplasmic protein, RseB. Under certain stress conditions, lipopolysaccharides (LPS) and outer membrane proteins (OMPs) are not incorporated into the outer membrane and accumulate in the periplasm. Periplasmic LPS binds RseB, freeing RseA to be cleaved by the OMP-activated protease DegS. This initiates further RseA degradation by the protease RseP, resulting in the release of RpoE into the cytosol (Barchinger & Ades, 2013; Lima *et al*, 2013). Over-expression of RseB down-regulates the RpoE pathway. In addition to this post-translational regulation, transcription of the *rpoE* gene is positively auto-regulated. It is highly likely that *H. influenzae* possesses a similar mechanism for the regulation of RpoE as in *E. coli*, although *rpoE* is essential in *E. coli* but not in *H. influenzae*. The overlapping effects on the transcriptome and phenotypes of the addition of beclomethasone, mutation of the sigma factor (*rpoE*) and mutation of the anti-sigma factor (*mclA*) genes are not consistent with a model in which glucocorticosteroids activate the RpoE stress response, but suggest they act to suppress the action of RpoE. Consistent with this contention, beclomethasone had no effect on the profile of outer membrane proteins of wild-type *H. influenzae* (Supplementary Fig S9). Suppression of RpoE action could involve direct binding of glucocorticosteroids to the sigma factor. To address this possibility, we determined the ability of purified RpoE to bind beclomethasone by isothermal titration calorimetry (Supplementary Fig S10). The experimental data show no binding and therefore do not support a direct binding model. These experiments do not rule out other mechanisms of beclomethasone action that include an inhibition of the regulated proteolysis of MclA/RseA or an influence on the RpoE::MclA balance by differential influences on transcription.

Our data show that the *H. influenzae rpoE* mutant biofilms were more tolerant of antimicrobial treatment than the wild-type. In contrast, *rpoE* mutants of other Gram-negative bacteria such as *Salmonella enterica* serovar Typhimurium and *Vibrio cholerae* have reduced survival in the presence of antimicrobials and attenuated virulence in various *in vitro* models (Humphreys *et al*, 1999; Osborne & Coombes, 2009). Furthermore, the *H. influenzae mclA* mutant biofilms showed similar tolerance to antibiotic treatment than the wild-type. These findings support the emerging view that biofilm formation in most bacteria instigates a completely different range of regulatory events to govern antimicrobial susceptibility than those activated during planktonic growth (Anderson *et al*, 2008; Osborne & Coombes, 2009).

Although the anti-inflammatory clinical benefits of glucocorticosteroid treatment are undeniable in many respiratory diseases, several recent studies have implicated such therapies in the development of bacterial pneumonia in asthma and COPD (Singanayagam *et al*, 2010). In addition, chronic bacterial infections of neutrophilic asthma airways that involve *H. influenzae* are connected to the development of airway disease that is steroid resistant (Essilfie *et al*, 2012). Our studies point to the need to consider the impact on bacterial behavior as one factor in the choice of which glucocorticosteroid to be used and in design of the treatment regime. For example, prednisolone triggered similar alterations in gene expression of *H. influenzae* to those seen with beclomethasone, whereas mometasone had little effect (Supplementary Fig S4). Would the use of mometasone therefore be preferential to other glucocorticosteroids for patients also being treated with azithromycin? Would stopping the glucocorticosteroid treatment before antibiotics are applied promote the antibacterial effect? While several clinical trials have reported an increased risk of bacterial pneumonia with the use of glucocorticosteroids in asthma and COPD patients, only specific patient trials designed to assess the above questions will inform clinicians. Overall, our data suggest the requirement for further studies to examine the action of glucocorticosteroids on bacteria that colonize the airway of individuals who rely on these therapeutic agents.

## Materials and Methods

### Bacterial strains, growth conditions and media

Strains and plasmids used in this study are described in Supplementary Table S4. *H. influenzae* strains were grown (overnight at 37°C) on brain–heart infusion agar plates supplemented with 10 μg/ml of hemin and 10 μg/ml of NAD (referred to as sBHI). *Escherichia coli* was grown on Luria-Bertani (LB) broth or LB agar plates at 37°C. When appropriate, the following concentrations of antibiotics were used: 50 μg/ml of kanamycin (Kan), 100 μg/ml of erythromycin (Em) and 150 μg/ml of azithromycin. Antibiotics were purchased from Sigma-Aldrich.

### DNA manipulations

Molecular biological methods such as isolation of plasmid and chromosomal DNA, PCR, plasmid transformation as well as restriction digestion were carried out using standard protocols (Sambrook *et al*, 1989). PCR products were cleaned using the PCR purification kit (Qiagen™), and DNA fragments were recovered from agarose gels using QIAquick minielute gel purification kit (Qiagen™). Oligonucleotide primers were purchased from Sigma-Genosys™.

### Construction of mutants in *H. influenzae* strains

Mutants in *H. influenzae* strains were constructed using a modified protocol of the one described previously (Morey *et al*, 2013). Genes *HI0628* and *HI0629* were amplified separately in two parts by PCR with Taq polymerase (Promega™) using Rd KW20 genomic DNA as the template. Primers were designed based on the genome sequence of *H. influenzae* Rd KW20 and detailed in Supplementary Table S5. The first part of each gene was amplified to include ∼200 bp of the region upstream of the predicted open reading frame, while the second part of the gene included ∼200 bp downstream of the predicted stop codon. As restriction sites external to these flanking regions, internal SmaI sites were incorporated onto each amplicon. The two separately amplified sequences were re-assembled in pBluescript and cloned into *E. coli* DH5a. Restriction digest using SmaI allowed the integration of an erythromycin cassette, which was taken from pBSLErm (Allen *et al*, 2005). The construct was linearized and used to transform chemically competent Rd KW20 using standard protocols. Transformants, which had successfully undergone recombination, were selected on sBHI containing 10 μg/ml Em. Complementation of mutant *H. influenzae* strains was carried out by inserting the relevant gene into open reading frame (ORF) HI0601.1; this ORF contains a frameshift in *H. influenzae* Rd KW20. The approach has been deployed successfully in a previous study (Morey *et al*, 2013). Copies of *HI0628* and *HI0629* genes were used to complement respective mutants (Supplementary Table S4).

### Construction of chromosomal reporter fusions

The protocol used for the construction of the *lux* reporter fusion for *HI1677* was a modification of the RED recombination protocols previously described by Lesic and Rahme (2008) and McCarthy *et al* (2010). The *HI1677* gene was amplified by PCR using forward and reverse primers HI1677-F and HI1677-R to include the region 250 bp upstream of the gene and was cloned into pGLuc. The *HI1677*::*lux* fusion was removed by restriction digest using HindIII and XbaI and cloned into pME6032-RedS cut with the same enzymes. This construct was electroporated into *H. influenzae* wild-type. Transconjugants were grown in sBHI to an optical density at 600 nm of 0.4 at 37°C, and recombination was induced by the addition of 0.2% L-arabinose for 1.5 h. The correct integration of the reporter cassette was confirmed by colony PCR using a reverse primer specific to the reporter and a forward primer specific to the upstream region of the target gene.

### Transposon mutagenesis and screening

A library of mutants in the *H. influenzae* strain carrying the *HI1677*::*lux* fusion was constructed using EZ::Tn<KAN-2> Tnp transposome (Epicentre technologies) as directed by the manufacturer. Briefly, 100 ng of transposon-containing plasmid was electroporated into newly prepared electrocompetent *H. influenzae* cells. Strains carrying the transposon insertion were identified by selection on Kan. The library of mutants was screened for loss of responsiveness of *HI1677::lux* expression to exogenous beclomethasone (50 μM). Strains were inoculated into microtiter wells containing sBHI medium with 50 μM beclomethasone by using a Qpix robot (Genetix™). The luciferase activity lysates of bacteria from each well were quantified as described previously (Deiwick *et al*, 1999). Briefly, equal amounts of bacterial cells as adjusted by the determination of optical density at 600 nm (OD600) were harvested by centrifugation and lysed. Luciferase activity in bacterial cell lysates was assayed using Luciferase Assay Kit (Promega™) and quantified in black microtiter plates by a Wallac Victor 21420 Multilabel Counter plate reader (Perkin Elmer™).

### Identification of transposon insertion sites

Genomic DNA was extracted from transposon mutants of interest as previously described (Sambrook *et al*, 1989). To identify the genes that were interrupted by the EZ::Tn transposon, the random amplification of transposon ends (RATE) PCR method of Ducey and colleagues (Ducey *et al*, 2005) was utilized. Amplicons were sequenced using the Inv-specific primers (Supplementary Table S5). Sequence data generated were examined with blastn and blastx (http://www.ncbi.nlm.nih.gov/BLAST/) software.

### Enrollment of subjects and sputum sample collection

Sputum samples from 24 asthma patients (January 2012–September 2013) were collected from Cork University Hospital. All study participants provided written consent. The Clinical Research Ethics Committee of the Cork Teaching Hospitals (CREC) granted full approval to the project. All sputa were analyzed and then frozen at −80°C in 1-ml aliquots for further study. Patient clinical parameters were also recorded including the participant’s age, lung function, pulmonary administered steroids or antibiotics, and colonization by microorganisms identified by standard clinical laboratory cultivation techniques.

### Ethics statement

Animal experiments were conducted in compliance with a protocol (# 16-051-11) approved by The Animal Experimentation Ethics Committee (AEEC) of University College Cork or Cork University Hospital. The Minister for Health accredits the University College Cork for conducting animal experiments. AEEC is guided by legislative requirements, in particular the Cruelty to Animals Act as amended and supplemented by the European Communities.

### Infection and treatment of animals

Mouse infection was performed with modification of the procedures described by Sekiya *et al* (2008) and Wu *et al* (1997). Four-week-old female C57BL/6 mice (Charles River) were injected intraperitoneally with cyclophosphamide at 3 days pre-infection and on the day of infection at a dose of 66 μg/g of body weight. Sample size was always five unless otherwise stated. Bacterial strains used for the intranasal challenge were grown in sBHI broth to an optical density (600 nM) of approximately 0.25. Subsequently, 20 μl of culture to have a final inoculum of 1 × 10^9^ colony-forming unit (CFU) was administered to each mouse. After every 24-h period, animals were treated with 100 μl of PBS or PBS containing beclomethasone (50 μM) was pipetted into the nares and involuntarily inhaled. Five mice were sacrificed by carbon dioxide asphyxiation at days 1, 3, 5 and 7 post-challenge. Bronchoalveolar lavage (BAL) fluid (100 μl) and blood (75 μl) were collected from each mouse. After exposure of the trachea, the nasopharynx was washed with 1 ml of buffer (0.5% trypsin, 0.02% EDTA in sterile PBS) by insertion of a 26-gauge needle sheathed in tubing into the tracheal end of the upper respiratory tract. Buffer was allowed to drip into the nasopharynx slowly and was collected from the nose, with each wash taking approximately 40 s. Both lungs and spleen were entirely removed, rinsed twice in PBS to remove excess blood, weighed and placed in 2 ml of sterile PBS. The lungs and spleen were then homogenized at 10,000 *g* for approximately 10 s. All blood, lung, spleen and BAL washout samples were then serially diluted and plated on agar to determine the number of viable bacteria. Total cells present in the BAL were counted, and a differential cell count was performed on cytospins stained with Diff Quick.

For animal experiments examining the effectiveness of azithromycin treatment against *H. influenzae* during respiratory infection, mice were intranasally inoculated with 20 μl of the bacterial suspension in PBS (1 × 10^8 ^CFU/mouse). Each mouse was administered azithromycin once daily over the course of infection. On day 3 after infection, the lung and spleen were removed, homogenized with PBS and plated on agar to determine the number of viable bacteria.

### RNA extraction

*H. influenzae* Rd KW20 strains (including mutants) were inoculated at an OD_600_ of 0.1 in sBHI [with 50 μM beclomethasone dipropionate (Sigma-Aldrich) if used]. Cultures were harvested during mid-log phase (OD_600_ = 0.7), and RNA was extracted using the High Pure RNA Isolation Kit (Roche). For the *in vivo* RNA samples, infected animals as described above were euthanized < 72 h post-infection. RNA was isolated from airway homogenate pellets using TRIzol according to the manufacturer’s instructions. Samples were treated with DNase, and then rRNA was removed from 1 to 5 μg of total RNA using the Ribo-Zero kit for Gram-negative bacteria (Epicentre). rRNA-depleted samples were concentrated by EtOH precipitation.

### Gene expression profiling experiments

RNA quality was assessed on a Bioanalyser PicoChip (Agilent), and RNA quantity was measured using the RNA assay on QuBit fluorometer (Life Technologies). Ribosomal RNA was depleted with Ribo-Zero™ rRNA Removal Kits for Gram-negative bacteria (Epicentre). The percentage of rRNA contamination was checked on a Bioanalyser PicoChip (Agilent).

The rRNA-depleted sample was processed using the Illumina TruSeq RNA v2 sample preparation kit. In brief, the sample was chemically fragmented to ∼200 nt in length and the cleaved RNA fragments were primed with random hexamers into first-strand cDNA using reverse-transcriptase and random primers. The RNA template was removed, and a replacement strand was synthesized to generate ds cDNA. The ds cDNA was end-repaired to remove the overhangs from the fragmentation into blunt ends. A single “A” nucleotide was added to the 3′ ends on the blunt fragments, which is complementary to a “T” nucleotide on the 3′ end of the Illumina adapters. At this stage, adapters containing 6-nt barcodes were used for different samples to allow the pooling of multiple samples together. The resulted bar-coded samples were enriched by 10 cycles of PCR to amplify the amount of DNA in the library. The final cDNA libraries were sequenced on an Illumina HiSeq2000 as per the manufacturer’s instructions.

The fluorescent images were processed to sequences using the Pipeline Analysis software 1.8 (Illumina). Raw sequence data obtained in Illumina FASTQ-format were first separated by their barcode sequence by comparing the first six bases with the expected barcode sequences. Successfully detected barcodes were removed from the sequence leaving paired-end reads of 30 nt in length, while reads containing no recognizable barcode sequence were discarded.

Reads for each sample were aligned to the *H. influenza*e Rd KW20 GCA_000027305.1 genome assembly (Ensembl bacteria genome database) using Bowtie version 2.0 with default parameters and randomness which when the program is faced with a sequence that aligns to multiple parts of the genome equally well, chooses one region randomly and the others are discarded. Transcript abundance was determined using the feature counts program to estimate the level of transcription for each gene, and the number of reads that mapped within each annotated coding sequence (CDS) was determined.

Differential expression was assessed using DESeq2, which estimates variance-mean dependence in read counts and uses negative binomial distribution to test for differential expression. The *P*-value for fold change is calculated and adjusted to remove the effects of repetition. The entire dataset has been deposited in the European Bioinformatics Institute (EBI) European Nucleotide Archive site under accession number ERG003569.

### Quantitative real-time PCR assays

The effect of *HI0628* or *HI0629* mutation or the addition of 50 μM of various steroids [beclomethasone dipropionate, prednisone, mometasone, dehydroepiandrosterone (Sigma-Aldrich)] to *H. influenza*e strains (including clinical isolates) on expression of genes was monitored by qRT–PCR. RNA was isolated from cultures of wild-type strain, wild-type supplemented with 50 μM steroid or mutant grown to an OD600 of 0.7, converted to cDNA using AMV Reverse Transcriptase (Promega) using conditions specified by the manufacturer. The quantitative PCR was carried out using Platinum® SYBR® Green qPCR SuperMix-UDG (Invitrogen). The primers used to amplify the genes are listed in Supplementary Table S2. As a control, RT–PCR was similarly applied to analyze expression of the 16S rRNA gene. The reverse transcription and PCR protocols were performed as described previously. The amplified products were subjected to electrophoresis on 2.5% agarose gels and stained with ethidium bromide. RT–PCR analysis was repeated at least twice for each gene tested.

### Cultivation and image analysis of biofilms

*H. influenzae* strains were allowed to form biofilm in static μ-well chambers (Ibidi-iTreat) containing sBHI media incubated at 37°C as previously described (Jurcisek *et al*, 2011). These chambers have a physically treated cycloolefin polymer exterior with a surface energy of around 72 mN/m. When required, steroid at a concentration of 1 or 10 or 50 μM was added during initial biofilm formation. Biofilm antibiotic susceptibility testing was carried out on 24-h-old biofilms of *H. influenzae* strains grown as described above (in the presence or absence of steroid as required) and then treated with 150 μg/ml azithromycin for 3 h before visualization and quantification.

Biofilms were stained and visualized using SYTO 9 to color live biofilm cells green and propidium iodide stain (Life Tech), a normally cell-impermeable stain, to color dead cells red. All microscopic observations and image acquisitions were performed on a Zeiss LSM780 confocal laser scanning microscope equipped with an argon–krypton laser and with detectors and filter sets for monitoring SYTO 9 and for the recording of reflection (light) images. Images were obtained using a 63×/1.4 Plan-APOChromat differential interference contrast objective or a 40×/1.3 Plan-Neofluor oil objective. Multichannel simulated fluorescence projection (SFP) images, vertical *xz* sections through the biofilms and simulated three-dimensional (3D) images were generated using the IMARIS software package (Bitplane). Biofilm images were obtained to quantify biomass as described previously using COMSTAT software.

### Statistical analysis

Significant differences between the means plus or minus standard deviations (SDs) of different groups were examined using a two-tailed unpaired Student’s *t-*test. A *P*-value of less than 0.05 was regarded as statistically significant. All variables remained significant after multiple testing.

## Supporting Information

**Supplementary Legends**

**Review Process File**
